# Transcriptome responses to heat- and cold-stress in ladybirds (*Cryptolaemus montrouzieri* Mulasnt) analyzed by deep-sequencing

**DOI:** 10.1186/s40659-015-0054-3

**Published:** 2015-11-19

**Authors:** Yuhong Zhang, Hongsheng Wu, Jiaqin Xie, Ruixin Jiang, Congshuang Deng, Hong Pang

**Affiliations:** State Key Laboratory of Biocontrol, School of Life Sciences, Sun Yat-sen University, Guangzhou, 510275 Guangdong China; Guangdong Entomological Institue, Guangzhou, 510260 Guangdong China

**Keywords:** Coccinellidae, Heat tolerance, Cold tolerance, Digital gene expression

## Abstract

**Background:**

Changed temperature not only threaten agricultural production, but they also affect individual biological behavior, population and community of many insects, and consequently reduce the stability of our ecosystem. Insect’s ability to respond to temperature stress evolved through a complex adaptive process, thus resulting in varied temperature tolerance among different insects. Both high and low extreme temperatures are detrimental to insect development since they constitute an important abiotic stress capable of inducing abnormal biological responses. Many studies on heat or cold tolerance of ladybirds have focused on measurements of physiological and biochemical indexes such as supercooling point, higher/lower lethal temperatures, survival rate, dry body weight, water content, and developmental duration. And studies of the molecular mechanisms of ladybird responses to heat or cold stress have focused on single genes, such as those encoding heat shock proteins, but has not been analyzed by transcriptome profiling.

**Results:**

In this study, we report the use of Digital Gene Expression (DGE) tag profiling to gain insight into transcriptional events associated with heat- and cold-stress in *C. montrouzieri*. About 6 million tags (49 bp in length) were sequenced in a heat stress group, a cold stress group and a negative control group. We obtained 687 and 573 genes that showed significantly altered expression levels following heat and cold shock treatments, respectively. Analysis of the global gene expression pattern suggested that 42 enzyme-encoding genes mapped to many Gene Ontology terms are associated with insect’s response to heat- and cold-stress.

**Conclusions:**

These results provide a global assessment of genes and molecular mechanisms involved in heat and cold tolerance.

## Background

With the impact of human activities on the climate, extreme temperature events are becoming more and more frequent. Fluctuations in environmental temperatures are encountered over the life span of most organisms. Many species have a metabolism that is adapted to the temperature range of the environment in which they evolved. When the external temperature out of this range, this triggers an evolutionarily conserved heat stress transcriptome response modulating genes that control multiple cellular activities including protein folding, protein degradation, transport, metabolism, DNA repair, and replocaion [1, 2].

Insects are relatively sensitive to temperature changes [3, 4]. Temperature has a direct impact on ontogenetic development, survival, and reproduction, while an indirect impact on generation time and population growth rate [5]. Both high and low extreme temperatures are detrimental to insect development since they constitute an important abiotic stress capable of inducing abnormal biological responses [6]. Insect’s ability to respond to temperature stress evolved through a complex adaptive process, thus resulting in varied temperature tolerance among different insects [7]. The ever-increasing occurrences of extreme weather events can impact natural predators in the field. Owing to such a difference in tolerance, temperature changes could consequently alter the synchrony between pests and their natural predators. For instance, if predators are relatively more sensitive to temperature changes than the pests, the latter will be able to escape from the control by the former. As a result, damages to crop plants incurred by the pests will be more severe, and furthermore, the predators might be driven to extinction [8]. It has been demonstrated that high temperatures are conducive to changes in insect metabolism, respiration, nervous and endocrine systems [9]. Insects respond to heat stress with increased expression of many genes including those encoding heat shock proteins, heat shock transcription factors, the hsr-omega protein and phosphoglucose isomerase [10–13]. Also, insects develop cold resistance through mechanisms including freeze tolerance, freeze avoidance and accumulation of polyols [14].

The ladybird *Cryptolaemus montrouzieri* Mulsant (Coleoptera: Coccinellidae) is a native species of Australia. The importance of *C. montrouzieri* as a biological control agent is expected to gain wider recognition due to concerns about over-reliance on insecticide usage. Many studies on heat or cold tolerance of ladybirds have focused on measurements of physiological and biochemical indexes such as supercooling point, higher/lower lethal temperatures, survival rate, dry body weight, water content, and developmental duration [15, 16]. So far studies of the molecular mechanisms of ladybird responses to heat or cold stress have focused on single genes, such as those encoding heat shock proteins, but has not been analyzed by transcriptome profiling.

In the few years since its initial application, the high-throughput sequencing (also called deep sequencing or Next Generation Sequencing; NGS) has become a powerful tool that allows the concomitant sequencing of millions of signatures to the genome and identification of specific genes and the abundance of gene expression in a sample tissue [17]. Previous transcriptome profiling studies, based on microarray data, which has been the most commonly used technology over the last decade, have some limitations as well because genes are represented by unspecific probe sets and, at low expression levels, they cannot be reliably detected. Sequencing-based methods generate absolute rather than relative gene expression measurements and avoid these inherent limitations of microarray analysis [18–21].

Recently, NGS technology has been adapted for transcriptome analysis because of the inexpensive production of large volumes of sequence data [22–25]. The next generation sequencing system developed by Solexa/Illumina [26], which is also referred to as Digital Gene Expression (DGE) tag profiling, allows identification of millions of short RNAs directly from mRNA and of differentially expressed genes without either the need to use bacterial clones or for prior annotations [27–29]. DGE tag profiling have dramatically changed the way that resistance-relevant genes in insects are identified because these technologies facilitate investigations on the functional complexity of transcriptomes [30, 31].

Using a Digital Gene Expression (DGE) tag profiling approach, we employed the Illumina HiSeq™ 2000 platform to perform a deep transcriptome analysis of *C. montrouzieri* to gain insight into the molecular mechanisms of ladybird responses to heat and cold stresses. This approach was suitable for investigating deep transcriptome variations in ladybirds and identified several loci with high transcription signals for not previously identified genes. Our results yielded sets of up-regulated and down-regulated genes in response to heat and cold stress and some genes, both related to heat and cold tolerance in ladybirds, are discussed. Furthermore, our analysis even obtained some novel heat/cold stressed relevant transcripts and, therefore, the benefit of better understanding of the molecular mechanism of heat and cold tolerance may result.

## Results

### Analysis of DGE libraries

To investigate the transcriptome responses to heat and cold stress in *C. montrouzieri*, the Solexa/Illumina’s DGE system was used to perform high throughput tag-sequencing analysis on ladybird adult libraries. We sequenced three DGE libraries, namely NC, HS and CS with insects collected 2 h following treatments at 25, 38 and 4 °C, respectively. Major characteristics of these three libraries were summarized in Table 1. Approximately a total of 6 million expressed sequence tags per library were obtained (submitted to the NCBI Short Read Archive [SRA] database, Accession No. SRR346079). Prior to mapping, these tag sequences from the reference transcripts database [32], adaptor tags, low quality tags and tags with one copy were filtered, producing approximately 6 million in total of clean sequence tags per library. The distribution of the total and distinct clean tag copy numbers showed highly similar tendencies in the three libraries. The HS library had the highest number of both clean and distinct clean tags. The other two libraries had similar counts. Moreover, the HS library showed the highest ratio of the number of distinct clean tags over total clean tags (1.01 %), and the CS library showed the lowest percentage of distinct high copy number tags (4.88 %). These data suggested that more genes were detected in the HS library than that in the other two libraries and more transcripts expressed at lower levels in the CS library. To estimate whether or not the sequencing depth was sufficient for the transcriptome coverage, the sequencing saturation was analyzed in the three libraries. The genes that were mapped by all clean tags and unambiguous clean tags increased with the total number of tags. When the number of sequencing tags reached 2 million, library capacity reached saturation (Fig. 1).

**Table 1:** Major characteristics of DGE libraries and tag mapping to the reference transcripts database

	NC		HS		CS	
	Distinct tag	Total tag	Distinct tag	Total tag	Distinct tag	Total tag
Raw data	120164	6134223	133704	5798954	117658	5901493
Tags containing N	678	1963	713	2119	606	2092
Adaptors	43	77	41	71	36	65
Tag CopyNum <2	68023	68023	75048	75048	65218	65218
Clean tag	51420	6064160	57902	5721716	51798	5834118
CopyNum >1	51420	6064160	57902	5721716	51798	5834118
CopyNum >5	23386	5984211	25732	5629564	23338	5753027
CopyNum >10	16051	5928384	17181	5564674	15665	5694782
CopyNum >20	10615	5848664	10970	5473325	10123	5613306
CopyNum >50	5526	5684688	5374	5295392	4920	5446060
CopyNum >100	3022	5507459	2885	5120118	2531	5277864
Tag mapping						
All mapping	23180	1365846	27457	1235061	23818	1030557
Unambiguous mapping	22967	1343506	27245	1224209	23620	1019908
Unknown tag	28240	4698314	30445	4486655	27980	4803561

All Mapping represents the number of all tags mapped to the reference transcripts database, Unambiguous Mapping represents the number of unambiguous tags mapped to the reference transcripts database, unambiguous tags indicate the tags matched only to one gene

**Fig. 1:** These three figures show the relationship between the number of detected genes and sequencing amount (total tag number). When the sequencing amount reaches 2 million, the number of detected genes almost ceases to increase

### Analysis of tag mapping

A basic reference tag database of *C. montrouzieri* containing 38,381 transcript sequences was prepared for tag mapping. Among these sequences, genes with a CATG site accounted for 23,774 (61.94 %). Also, all CATG+ 17-base tags were used as gene’s reference tags. Finally, a total of 54,293 tag sequences, among which 53,872 (99.22 %) possessed an unambiguous match to reference tags were obtained. Based on aforementioned criteria, 45.08–47.42 % of the distinct clean tags were mapped to the virtual transcripts database, 44.67–47.05 % of the distinct clean tags were mapped unambiguously to the transcripts, and 52.58–54.92 % of the distinct clean tags did not map to the transcripts tag database (Table 1). The occurrence of unknown tags was probably due to factors such as the lack of ladybird genome sequences, incomplete *Nla*III digestion of cDNA during library preparation, many tags matching with noncoding RNAs and alternative use of polyadenylation signals and/or splicing sites [33, 34]. Solexa/Illumina sequencing can distinguish transcripts originating from both DNA strands. Based on the strand specificity of the sequencing tags obtained, bidirectional transcription was found in 10,156 to 11,420 of all detectable transcripts, including 8983 to 10,304 sense-strand transcripts and 5157 to 5519 antisense-strand transcripts (Table 2). In other words, the ratio of sense to antisense strands of the transcripts was approximately 1.8:1 for all the libraries. This suggests that, in spite of the high number of sense and antisense mapping events detected, the transcriptional regulation in the heat and cold response acts most strongly on the sense strand in ladybirds.

**Table 2:** Statistics of distinct tag mapping to gene (sense and antisense)

	NC		HS		CS	
	Number of genes	Percent	Number of genes	Percent	Number of genes	Percent
Clean tag	38381		38381		38381	
Perfect match (sense)						
1 tag → 1 gene	8629	22.48	9943	25.91	9089	23.68
1 tag → n gene	190	0.50	217	0.57	219	0.57
1 bp MisMatch (sense)						
1 tag → 1 gene	1219	3.18	1358	3.54	1151	3.00
1 tag → n gene	96	0.25	101	0.26	97	0.25
Perfect match (antisense)						
1 tag → 1 gene	5122	13.35	5311	13.84	4965	12.94
1 tag → n gene	76	0.20	74	0.19	66	0.17
1 bp MisMatch (antisense)						
1 tag → 1 gene	567	1.48	575	1.50	490	1.28
1 tag → n gene	26	0.07	26	0.07	12	0.03
All tag mapping to sense gene	8983	23.40	10304	26.85	9464	24.66
Unambiguous tag mapping to sense gene	8836	23.02	10145	26.43	9295	24.22
All tag mapping to antisense gene	5331	13.89	5519	14.38	5157	13.44
Unambiguous tag mapping to antisense gene	5285	13.77	5468	14.25	5116	13.33
All tag mapping to gene (sense and antisenese)	10156	26.46	11420	29.75	10600	27.62
Unambiguous tag mapping to gene (sense and antisense)	10016	26.10	11259	29.33	10441	27.20

### Identification of differentially expressed (DE) genes across treatments

Global analysis of transcriptome variations in *C. montrouzieri* adults exposed to each temperature treatment revealed the up- or down-regulation of genes transcribed between differential temperature points (HS/NC, CS/NC) across treatments. To compare the DE genes between libraries, the level of gene expression was determined by converting the number of unambiguous tags in each library to Tags Per Million (TPM). Out of all tag-mapped genes, 6859, 7925 and 7232 genes could be annotated by the NCBI non-redundant (Nr) database (E-value ≤ 10^−5^) in NC, HS and CS libraries, respectively. In order to find the significant changes in gene expression under heat and cold stresses, the DGE analysis with tags from these three groups was carried out based on Bayesian algorithm [35]. False discovery rates (FDR) ≤0.001 and the absolute value of the log_2_ Ratio ≥1 were used as a threshold to judge the statistical significance of gene expression. From the three data sets, 687 genes, mapped by a total of 2585 significantly changed tag entities, were detected in the HS/NC libraries, while the total number of genes (573) mapped by 2084 tag entities in the CS/NC libraries was a little lower. As compared to the NC data set, most of the genes (403) were up-regulated in the HS group, and most of the genes (389) were down-regulated in the CS group (Fig. 2). In the HS/NC and CS/NC libraries, we found 541 (78.75 %) and 432 (75.39 %) genes could be annotated by the Nr database; while no homologues for the other 146 (21.25 %) and 141 (24.61 %) genes were found. The top 20 most DE genes with Nr annotation in HS/NC and CS/NC libraries, respectively, are presented in Table 3. The most DE genes in the HS/NC group were those encoding small heat shock protein 21 (HSP21), keratin type I cytoskeletal 9 (KIC9) and Iris-A (IA), while that in the CS/NC group were those encoding HSP21, the vacuolar protein sorting (VPS) and the LIM protein (LIMP). Among the most DE genes, we noticed that 4 out of 20 genes appeared in both HS/NC and CS/NC groups including HSP21, KIC9, LIMP and AW1 (ATPase WRNIP1-like). All of them are most likely involved in both heat and cold tolerance. In addition, 5 HSPs out of 20 genes were found in HS/NC pairs, 29 HSPs and heat shock factor (HSFs) genes identified among all the HS/NC DE genes. These findings strongly suggest that HSPs and HSFs play an important role in regulating heat stress response at the gene expression level.

**Fig. 2:** Differential expression analyses of genes by DGE. ‘Not DEGs’ indicates ‘not detected expression genes’. For Figures **a** and **b**, the x-axis contains Log_10_ of transcript per million of the NC group and the y-axis indicates Log_10_ of transcript per million of the AS or CS groups. Limitations are based on FDR ≤0.001, and the absolute value of log_2_ Ratio ≥1

**Table 3:** Top most differentially expressed annotated genes between the HS/NC and CS/NC libraries based on the expressed tag frequency

Gene ID	log_2_ ratio (HS/NC < TPM >)	Annotation
HS/NC		
Locus_37579	7.60279	Small heat shock protein 21 isoform 1
Locus_2923	5.1454	Keratin, type I cytoskeletal 9
Locus_4481	4.82484	Iris-A
Locus_12479	4.74705	GE15901
Locus_11470	4.6968	Lethal(2) essential for life protein, l2efl
Locus_23537	4.36988	Small heat shock protein 21
Locus_3017	4.34878	Starvin CG32130-PE
Locus_930	4.12676	Glycine cleavage system h protein
Locus_35805	4.0602	GF23659
Locus_271	3.7271	LIM protein
Locus_25582	3.62017	Heat shock protein 70 cognate
Locus_1875	3.51019	Proline oxidase
Locus_13246	3.37113	GA19677
Locus_1446	3.37113	Thymosin beta isoform 2
Locus_27531	3.37113	Kelch-like 24
Locus_372	3.36106	Heat shock protein 1
Locus_927	3.29323	ATPase WRNIP1-like
Locus_15572	3.29323	Translation initiation factor eIF-2B subunit epsilon
Locus_387	3.27879	Heat shock protein 70
Locus_7854	3.25252	GA10992-PA
CS/NC		
Locus_37579	3.34239	Small heat shock protein 21 isoform 1
Locus_15315	3.30212	Vacuolar protein sorting
Locus_271	3.26394	LIM protein
Locus_232	3.24715	GI19648
Locus_927	2.91271	ATPase WRNIP1-like
Locus_16433	2.89616	Hypothetical UPF0293 protein
Locus_13581	2.75651	Transmembrane protein 205
Locus_1903	2.75435	UK114
Locus_8436	2.72052	39S ribosomal protein L36
Locus_2882	2.69502	LOC733269 protein
Locus_1270	2.65951	Casein kinase II beta subunit
Locus_28730	2.64807	Deoxyribodipyrimidine photo-lyase
Locus_6998	2.63977	KIAA0090 isoform 1
Locus_25474	2.6171	Nucleoporin 160 kDa
Locus_23418	2.5153	DNA-directed RNA polymerase I subunit RPA1
Locus_2871	2.46285	GF22743
Locus_2923	2.43676	Keratin, type I cytoskeletal 9
Locus_2576	2.3944	GG12605
Locus_17282	2.37627	Adapter-related protein complex 2 alpha 2 subunit
Locus_11450	2.29917	eIF2B- CG10315-PA

### Gene functional annotation in heat and cold stressed ladybirds

A GO analysis of DE genes in HS/NC and CS/NC pairs were performed by mapping each DE gene to GO terms (http://www.geneontology.org/), 41 GO terms were found in biological process categories. Under these categories, those related to metabolic, primary metabolic, cellular, biosynthetic and cellular metabolic processes were abundant in the DE genes. Specifically, 35 and 27 of the DE genes were categorized as gene responses to stimulus, and 27 and 19 of the DE genes were categorized as gene responses to stress in HS/NC and CS/NC pairs, respectively (Fig. 3).

**Fig. 3:** Gene classification based on gene ontology (GO) for differentially expressed genes in HS/NC and CS/NC libraries. The y-axis and x-axis indicate the names of clusters and the number of genes in each cluster, respectively. Only the biological processes were used for GO analysis

Functional annotation of DE genes was performed to map all the genes to terms in the KEGG database. We compared DE genes with the whole transcriptome background in order to search for genes involved in metabolic or signal transduction pathways that were significantly enriched. Among all the DE genes between HS/NC and CS/NC data sets, 379 and 309 genes were mapped in 173 and 165 terms in the KEGG pathway database, respectively. Notably, specific enrichment of genes was observed for the KEGG pathway with a significant *P* value of <0.05 indicating involvement in both heat and cold response metabolic or signal transduction pathways (Table 4). These genes were also involved in drug metabolism (other enzymes, metabolic pathways, metabolism of xenobiotics by cytochrome P450 and drug metabolism), cytochrome P450, antigen processing and presentation, starch and sucrose metabolism, steroid hormone biosyntheses, retinol metabolism, amino sugar and nucleotide sugar metabolism, oxidative phosphorylation, tyrosine metabolism and fatty acid metabolism. However, some other pathways were only influenced under heat stress, such as protein processing in the endoplasmic reticulum, ribosomes, NOD-like receptor signaling pathways, neuroactive ligand-receptor interaction, fatty acid elongation in mitochondria, insect hormone biosynthesis, cardiac muscle contraction, the PPAR signaling pathway and complement and coagulation cascades. Some other pathways were only affected under cold stress, such as ascorbate and aldarate metabolism, other glycan degradation, phagosome, alpha-linolenic acidmetabolism, pentose and glucuronte interconversions, linoleic acid metabolism and glycerolipid metabolism.

**Table 4:** Pathway enrichment analysis for DE genes

No.	Pathway ID	Pathway	Number of DE genes	P-value
HS/NC				
1	ko04612	Antigen processing and presentation	18	1.45E−11
2	ko04141	Protein processing in endoplasmic reticulum	28	1.01E−07
3	ko03010	Ribosome	14	1.57E−06
4	ko00983	Drug metabolism—other enzymes	18	2.15E−05
5	ko01100	Metabolic pathways	88	6.79E−05
6	ko00140	Steroid hormone biosynthesis	13	0.000282
7	ko00830	Retinol metabolism	13	0.00053
8	ko00520	Amino sugar and nucleotide sugar metabolism	10	0.000747
9	ko04621	NOD-like receptor signaling pathway	7	0.001046
10	ko00190	Oxidative phosphorylation	11	0.002814
11	ko04080	Neuroactive ligand-receptor interaction	12	0.003165
12	ko00980	Metabolism of xenobiotics by cytochrome P450	12	0.004002
13	ko00982	Drug metabolism–cytochrome P450	12	0.004793
14	ko00062	Fatty acid elongation in mitochondria	3	0.006405
15	ko00860	Porphyrin and chlorophyll metabolism	9	0.007187
16	ko00981	Insect hormone biosynthesis	4	0.009516
17	ko00500	Starch and sucrose metabolism	10	0.011378
18	ko04260	Cardiac muscle contraction	11	0.015768
19	ko03320	PPAR signaling pathway	7	0.026265
20	ko04610	Complement and coagulation cascades	6	0.029497
21	ko00350	Tyrosine metabolism	7	0.032871
22	ko00071	Fatty acid metabolism	5	0.044768
CS/NC				
1	ko00983	Drug metabolism—other enzymes	23	3.61E−10
2	ko01100	Metabolic pathways	91	5.30E−10
3	ko04142	Lysosome	26	7.61E−09
4	ko00980	Metabolism of xenobiotics by cytochrome P450	19	2.03E−08
5	ko00982	Drug metabolism—cytochrome P450	19	2.94E−08
6	ko04612	Antigen processing and presentation	13	5.57E−08
7	ko00500	Starch and sucrose metabolism	16	4.56E−07
8	ko00140	Steroid hormone biosynthesis	15	1.56E−06
9	ko00830	Retinol metabolism	15	3.55E−06
10	ko00520	Amino sugar and nucleotide sugar metabolism	12	5.03E−06
11	ko00053	Ascorbate and aldarate metabolism	10	7.59E−05
12	ko00511	Other glycan degradation	5	9.30E−05
13	ko00190	Oxidative phosphorylation	12	0.000137
14	ko04145	Phagosome	17	0.000231
15	ko00592	Alpha-Linolenic acid metabolism	9	0.000329
16	ko00860	Porphyrin and chlorophyll metabolism	10	0.000471
17	ko00040	Pentose and glucuronate interconversions	9	0.001679
18	ko00350	Tyrosine metabolism	8	0.003413
19	ko00591	Linoleic acid metabolism	7	0.003593
20	ko00561	Glycerolipid metabolism	9	0.004786
21	ko00071	Fatty acid metabolism	6	0.004981

### Validation of DGE data by QPCR

To validate the differential DGE results identified by Solexa/Illumina sequencing, we selected 12 genes for quantitative RT-PCR confirmation. The gene set included 4 down-regulated genes (cytochrome p450 [P450], acyl carrier protein[ACP], serine protease P80[SP80] and chitinase 3 [CHI3]) and 8 up-regulated genes (novel protein zgc[NPZ], macrophage-stimulating protein receptor[MSPR], NTF2, ATPase WRNIP1[AW1], heat-responsive protein 12 [HRP], casein kinase beta polypeptide [CKBP], stress-induced-phosphoprotein 1 [SIP1] and ribose-phosphate pyrophosphokinase [RPP]). Results from HS and CS samples were presented as fold changes in gene expression normalized to the house keeping (beta-tubulin) gene and relative to the NC sample. Although the absolute fold changes differed between qPCR and DGE analysis, the direction of change was concordant for each gene (Fig. 4).

**Fig. 4:** Six differentially expressed genes have been identified by qRT-PCR, including HRP, CKBP, SIP1, RPP, P450 and CHI3. The left y-axis indicates the relative expression level by qRT-PCR, and the right y-axis indicates the log_2_ Ratio of NC, HS and CS libraries by DGE

## Discussion

*C. Montrouzieri* is mainly distributed in the subtropical and tropical regions, it generally suitable for the survival temperature in 20–30 °C, although the different climate make it a certain regional group differences. Heat and cold tolerance of *C. montrouzieri* directly limits its adaptation to climatic changes and distribution. Since *C. montrouzieri* is one of the major natural enemies of mealybugs, such tolerance to extreme temperatures would have significant effects and ramifications on pest control. Previous studies on tolerance of *C. montrouzieri* to extreme temperatures showed that, high temperatures (32–36 °C) killed all larvae and pupae, and stopped the adults from laying eggs, while at 40 °C, the adults stopped feeding and 40 % of them died [13]. Low-temperature treatment at 10 °C stopped the adults from feeding, treatment at 2 °C suspended their movement, and 40 % of the adults died when temperature raised slowly from −2 °C to above 15 °C. Our previous observation (unpublished data) also revealed that high-temperature treatment at 38 °C or low-temperature treatment at 4 °C for 12 h would not cause death of *C. montrouzieri*, but extended treatment to 48 h would kill almost half of the Tested sample population. We chose these two temperatures because such temperatures can rapidly stimulate stress responses while treatment at such temperatures for 2 h would not cause lethal cell damage or organ failure. Development of tolerance to extreme temperatures by *C. montrouzieri* is likely through their avoidance behavior and expression regulation of several tolerance-related proteins and metabolisms. Comprehensive investigation of gene expression regulation under heat and cold stress will be of great importance in order to understand the biochemical and physiological adaptation process in *C. montrouzieri*, since there are only 62 *Cryptolaemus* sequence entries in GenBank. Previous transcriptome profiling studies using microarray data analysis, which has been the most commonly used technology over the last decade, provided limited information because many genes are under-represented by unspecific probe sets and relatively low expression levels for reliable gene detection. Sequencing-based methods generate absolute rather than relative gene expression measurements and avoid such inherent limitations as found in microarray data analysis [18, 21]. In this study, large-scale DGE tag data were obtained by high throughput sequencing to provide a clear insight into the molecular mechanism of the response to temperature stress in *C. montrouzieri*.By targeting a defined cDNA library, the DGE method can generate broader transcriptome coverage and a higher number of cDNA tags per gene, leading to more precise gene transcription information. Provided that a reference genome or transcriptome database is available and that the aim is to quantify transcript levels between different biological samples, this method is perfectly suited for deep transcriptome analysis [36].

In contrast to many previous studies on transcriptome analysis using mixed samples, we chose adult samples based on the premise that adult period is the longest part of the life cycle of *C. montrouzieri* and the adults also have the strongest tolerance to extreme temperatures. It is in adult form that the *C. montrouzieri* passes through winter and lays eggs when temperature rises to appropriate levels. A mixed sample of ladybirds at all stages may provide more sequence data, but such data may render the differentially expressed genes less obvious. In addition, for non-model insects such as *C. montrouzieri*, analysis of differentially expressed genes in adults can improve the accuracy to detect temperature tolerance-related genes compared to analysis of mixed samples. Although sequencing the mixed mRNAs was lack of correlation analysis, the results of the group change tendency is still representative.

We sequenced 3 distinct cDNA libraries obtaind from a heat-stressed group, a cold stressed group and a negative control group, using the DGE method. we obtained 10,016 to 11,259 (among three libraries) tag-mapped genes out of 38,381 transcripts (26.10–29.33 %) by mapping the tags to a transcriptome reference database. Many transcripts did not map to tags, most likely as a result of differences in gene expression at different development ladybird stages, distinct genes might be matched by the same tags and were possibly removed from the data sets, and/or a CATG site does not exist in all genes. In our transcriptome database, 14,607 genes (38.06 %) without CATG sites could not generate 49 bp tags to sequence on the Solexa/Illumina platform. In addition, more than 52 % (NC: 54.92 %, HS: 52.58 %, CS: 54.01 %) of the distinct clean tags could not be mapped to the transcriptome reference database. The occurrence of unknown tags was most likely due to the lack of ladybird genome sequences, the incomplete *Nla*III digestion during library preparation, many tags matching noncoding RNAs and the usage of alternative polyadenylation and/or splicing sites [33, 34].

Recently, some other species transcriptome response to temperature stress were reported, and they almost interest in species response to heat stress, such as chicken, marine snail, duck, fungus, etc. [37–40]. However numbers of the regulated genes were very different in different animal, many same biological processes and pathways were found by differential expression genes, including transcription factor, chromatin modification, signaling pathways, DNA repair and replication, translation, ect. In this study, stress by heat and cold treatments resulted in significant alterations of transcriptome profile in the ladybird, including change in expression of 1033 transcripts. Among them, 227 genes were affected by both heat and cold stresses, including 42 significantly differentially transcribed enzyme-related gene (Fig. 5). Fifteen genes were strongly up-regulated by heat and cold stress, including those encoding carboxylesterase, juvenile hormone esterase, mps one binder kinase, cathepsin, ATP synthase, beta-ureidopropionase, phosphatidylinositol-3,4,5-trisphosphate 3-phosphatase, RNA helicase, beta-1,4-mannosyltransferase, ribose-phosphate pyrophosphokinase, endonuclease-reverse transcriptase and casein kinase. Based on the finding that genes encoding multiple serine proteases, cytochrome, cathepsin, chitinase and some other enzymes were down-regulated (Fig. 5), we speculated that these enzymes are most likely relevant to both heat and cold tolerance.

**Fig. 5:** Enzymes differentially transcribed in ladybirds stressed by heat and cold. Clustering analysis based on transcription levels was performed on 42 enzyme-encoding genes showing differential transcription in *C. montrouzieri* exposed to heat and cold. *Color scale* from *red* to *green* indicates Log_2_ transcription ratios from +2 (fourfold over transcription) to −2 (fourfold under transcription). For each gene, gene ID and annotation are indicated

However, these significantly differentially transcribed enzyme-related genes represented only a small proportion of the total transcripts that were found in transcriptome database. In addition to these annotated genes, 146 and 141 genes out of HS/NC group and CS/NC group, respectively, could not be matched with any existing genes. Novel genes that may be involved in the insecticide response might be identified from this group in the future.

## Methods

### Experimental insect and sample preparation

Stock cultures of *C. montrouzieri* were reared on mealybugs (*Planococcus citri* Risso) at Sun Yet-Sen University, Guangzhou, China, and were maintained in laboratory for more than 10 years before the onset of this project. *C. montrouzieri* adults (3 days after eclosion of female adults) were obtained by rearing the colony under insectary conditions at 25 ± 1 °C and with a photoperiod of 14 h light and 10 h darkness. To understand the transcriptome responses to extreme temperatures, two groups named heat stress group (HS) and cold stress group (CS) were treated at 38 and 4 °C for 2 h, respectively. In addition, a negative control group (NC) without temperature stress was treated at 25 °C for 2 h. Finally, these samples were harvested and immediately frozen in liquid nitrogen for subsequent analysis.

### RNA extraction, DGE library construction and sequencing

Total RNA was extracted from each sample group using the UNlQ-10 Column Trizol Total RNA Isolation Kit (Sangon, Shanghai) according to the manufacturer’s instructions. The integrity of RNA samples was determined using a 2100 Bioanalyzer (Agilent Technologies) and standardized with a minimum RNA integrated number value of 7.5. For each group, total RNA from 3 replicates was pooled together in equal quantities. Approximately 6 μg of RNA representing each group were used for Solexa/Illumina sequencing.

Sequencing tag library construction was performed in parallel using an Illumina Gene Expression Sample Prep Kit. Briefly, mRNA was isolated from total RNA using magnetic oligo (dT) beads. First and second strand cDNA were synthesized, and bead-bound cDNA was subsequently digested with the restriction enzyme *Nla*III, which recognizes and cleaves at the CATG site. Then the 3′-cDNA fragments attached to oligo (dT) beads were ligated to Illumina Adapter 1, which contained a recognition site for the restriction enzyme *Mme*I for cleavage 17 bp downstream of the CATG site to produce tags with adapter 1. After removing the 3′ fragments via magnetic bead precipitation, the Illumina adaptor 2 was ligated to the 3′ ends of tags, rsulting in tags with different adaptors attached to both ends to form a tag library. After 15 cycles of linear PCR amplification, 95 bp fragments were purified by 6 % TBE PAGE gel electrophoresis. Subsequently, the single-chain molecules were fixed onto the Illumina Sequencing Chip (flow cell). Each molecule was allowed to grow into a single-molecule cluster sequencing template through in situ amplification. In this process, color-labeled nucleotides were added, and products were sequenced via the method of sequencing by synthesis (SBS). Up to millions of sequence reads with a length of 49 bp were generated. The Illumina Sequencing of three libraries for each of HS, CS and NC groups was performed by Beijing Genomics Institute (BGI), Shenzhen, China. The raw data (tag sequences) were submitted to the NCBI SRA database with the accession number SRR346079.

### DGE tag profiling

For the raw data, we filtered all raw sequence reads by the Illumina pipeline. All low quality tags, such as tags with unknown sequences ‘N’, empty tags (sequences with only adaptor sequences), low complexity, and tags with only one copy (probably resulting from sequencing errors) were removed, then the remainder of tags are clean tags. For annotation, a virtual library containing all the possible CATG + 17 base length sequences were created using a reference transcripts database [32] (assembled by our laboratory, and the raw data was deposited in the NCBI SRA database with the Accession No. SRR343064) by SOAP programs (developed by Beijing Genomics Institute, Beijing, China). If a clean tag were mapped to a gene in virtual library, the number of this tag was considered to be the expression of the gene. For monitoring the mapping events on both strands, both the sense and complementary antisense sequences were included in the data collection. All clean tags were mapped to the virtual library and only one nucleotide mismatch was allowed. Clean tags that could be mapped to reference sequences in virtual library were filtered from multiple genes. The remainders of the clean tags were designed as unambiguous clean tags. For gene expression analysis, the number of unambiguous clean tags for each gene was calculated and then normalized to the number of transcripts per million clean tags (TPM) [20, 41], and the differentially expressed tags were used for mapping and annotation.

### Gene expression pattern analysis

A statistical analysis of the frequency of each tag in these three cDNA libraries was performed to compare gene-expression results. Statistical comparison was performed with custom written scripts using the method described by Audic and Claverie [35]: Denote the number of unambiguous clean tag from gene A as x, as every gene’s expression occupies only a small part of the library, the p(x) is in the Poisson distribution.

$$p(x) = \frac{{e^{ - \lambda } \lambda^{x} }}{x!}$$

where λ is the real transcripts of the gene.

The total clean tag number of the sample 1 is N1, and total clean tag number of sample 2 is N2; gene A holds x tags in sample 1 and y tags in sample 2. The probability of gene A expressed equally between two samples can be calculated with:

$$\begin{aligned} 2\sum\limits_{i = 0}^{i = y} {p(i|x)} \hfill \\ {\rm or} \, 2 \times \left( {1 - \sum\limits_{i = 0}^{i = y} {p(i|x)} } \right)\;\;\left( {if\;\sum\limits_{i = 0}^{i = y} {p(i|x)} > 0.5} \right) \hfill \\ p(y|x) = \left( {\frac{{N_{2} }}{{N_{1} }}} \right)^{y} \frac{(x + y)!}{{x!y!\left( {1 + \frac{{N_{2} }}{{N_{1} }}} \right)(x + y + 1)}} \hfill \\ \end{aligned}$$

The P value corresponds to the DGE test. The false discovery rate (FDR) is a method to determine the threshold of the P value in multiple tests and analyses through manipulating the FDR value. We used “FDR ≤ 0.001 and the absolute value of log_2_ Ratio ≥1” as the threshold to judge the significance of gene expression differences. The Nr protein database with an E-value cut-off of 10^−5^ was used for a blast search and annotation by BLASTx using Blast2GO software. In gene expression profiling analysis, GO enrichment analysis available at the Gene Ontology Consortium website http://www.geneontology.org was performed using a hypergeometric test to map all DGEs to terms in the GO database with a corrected P-value ≤0.05. For pathway enrichment analysis, we mapped all differentially expressed genes to terms in the KEGG database and identified significantly enriched KEGG terms relevant to extreme temperatures with P-value ≤0.05 and Q-value ≤0.05. We also performed cluster analysis of DGE patterns using software programs Cluster [42] and Java Treeview [43].

### Quantitative RT-PCR analysis

To verify DGE analysis results, we designed 12 pairs of primers using Primer Premier 5.0 to perform qPCR analysis targeting 8 up-regulated and 4 down-regulated genes. Beta-tubulin used as the house keeping gene due to its stable expression in NC/HS/CS group in this study. The RNA samples used for the qPCR assay were the same as that used in the DGE experiments with independent RNA extractions from three replicates. The first cDNA strand was synthesized from 1.0 μg of total RNA by a PrimeScript RT reagent Kit (TaKaRa). The qPCR was performed using a cycling program of 95 °C for 30 s, and 40 cycles of 95 °C for 10 s, 55 °C for 10 s and 72 °C for 20 s on an iQ™ 5 Multicolor real-time PCR detection system (Bio-RAD). With the application of SYBR Premix Ex Taq polymerase (TaKaRa, Ohtsu, Japan) and SYBR-Green detection method was followed, according to manufacturer’s instructions. The forward and reverse primers used for qPCR are shown in Table 5. Each reaction was run in triplicate. After amplification the average threshold cycle (C_t_) was calculated for each sample. The beta-tubulin gene was used as a reference to normalize expression levels, and the relative expression levels of genes were calculated by the $2^{{ - \Delta \Delta C_{t} }}$ method.

**Table 5:** Primers used for validation analysis

Gene name	Gene ID	Primer
Heat-responsive protein 12	Locus_1903	5′-TTATCCAAACCGAGAACACCG-3′
		5′-GAATGTGCTCCGAAACCTGTG-3′
Casein kinase beta polypeptide	Locus_1270	5′-TGGGTTTATCTGATGTTCCTGG-3′
		5′-CGGTATGATGGTGACGTGATG-3′
Stress-induced-phosphoprotein 1	Locus_1379	5′-GTATGGAAACTGCCGGTATTGG-3′
		5′-GCGGGATCTCTAAGTATTTGTTGC-3′
Ribose-phosphate pyrophosphokinase	Locus_1071	5′-AGGCTTAACGTCGAGTTTGCC-3′
		5′-GTCCTTGACATCTCCCACTAATACC-3′
Cytochrome p450	Locus_2703	5′-CATGGTTCACAGCGTGTAATAGC-3′
		5′-GTGCCTTAGGCAAACGTCAAAT-3′
Chitinase 3	Locus_53	5′-GACACTATGCACCTCTGAACGC-3′
		5′-CCAGTAAGTGATACCTCGGAAAAC-3′
Novel protein zgc 112389	Locus_15691	5′-TTTAGGTTCTCCACTATGGCTAC-3′
		5′-AGTAATCACAGCAACAGCCAAT-3′
Serine protease P80	Locus_10683	5′-TTTGAAACTCGAAAGGGCATTG-3′
		5′-GAATAGGATAGACGAGCAAGG–3′
NTF2	Locus_15496	5′-AAAGGAGACACTTAATTTCCAGG-3′
		5′-TCCCATTACACCATTACCATTC-3′
Macrophage-stimulating protein receptor	Locus_23091	5′-TTTCTCGTGGGACAAGATTACC-3′
		5′-GAGTCTCGCAGTTAGGTCTTTCAC-3′
Acyl carrier protein	Locus_2931	5′-ATTCGCTGGATCATGTTGAAGT-3′
		5′-GCTTCTCAGCATCGGCATCT-3′
ATPase WRNIP1	Locus_927	5′-CTGAGGCTTCTCCTGCTAAACG-3′
		5′-CCATTCAAGGCAGGCGATTT-3′
Beta-tubulin	Locus_627	5′-CACGGAAGGTACTTGACTGTTG-3′
		5′-GCTGCTGTTCTTGTTTTGGATG-3′

## References

[1] Feder ME, Hofmann GE (1999). Heat-shock proteins, molecular chaperones, and the stress response: evolutionary and ecological physiology. Annu Rev Physiol.

[2] Kregel KC (1985). Heat shock proteins: modifying factors in physiological stress responses and acquired thermotolerance. J Appl Physiol.

[3] Deutsch CA, Tewksbury JJ, Huey RB, Sheldon KS, Ghalambor CK, Haak DC (2008). Impacts of climate warming on terrestrial ectotherms across latitude. Proc Natl Acad Sci USA.

[4] Gillooly JF, Brown JH, West GB, Savage VM, Charnov EL (2001). Effects of size and temperature on metabolic rate. Science.

[5] Forster J, Hirst AG, Woodward G (2011). Growth and development rates have different thermal responses. Am Nat.

[6] Kang L, Chen B, Wei JN, Liu TX (2009). Roles of thermal adaptation and chemical ecology in Liriomyza distribution and control. Annu Rev Entomol.

[7] Piiroinen S, Lyytinen A, Lindstrom L (2013). Stress for invasion success? Temperature stress of preceding generations modifies the response to insecticide stress in an invasive pest insect. Evol Appl.

[8] Sinclair BJ, Addo-Bediako A, Chown SL (2003). Climatic variability and the evolution of insect freeze tolerance. Biol Rev Camb Philos Soc.

[9] Garcia SL, Rodrigues VL, Garcia NL, Ferraz Filho AN, Mello ML (1999). Survival and molting incidence after heat and cold shocks in Panstrongylus megistus Burmeister. Mem Inst Oswaldo Cruz.

[10] Solomon JM, Rossi JM, Golic K, McGarry T, Lindquist S (1991). Changes in hsp70 alter thermotolerance and heat-shock regulation in Drosophila. New Biol..

[11] Morgan TJ, Mackay TF (2006). Quantitative trait loci for thermotolerance phenotypes in Drosophila melanogaster. Heredity..

[12] Rank NE, Bruce DA, McMillan DM, Barclay C, Dahlhoff EP (2007). Phosphoglucose isomerase genotype affects running speed and heat shock protein expression after exposure to extreme temperatures in a montane willow beetle. J Exp Biol..

[13] Chen J, Kitazumi A, Alpuerto J, Alyokhin A, de Los Reyes B (2015). Los Reyes B. Heat-induced mortality and expression of heat shock proteins in Colorado potato beetles treated with imidacloprid. Insect Sci..

[14] Salin C, Vernon P, Vannier G (2003). Cold resistance in the lesser mealworm *Alphitobius diaperinus* (Panzer) (Coleoptera: Tenebrionidae). Cryo Letters..

[15] Rank NE, Bruce DA, McMillan DM, Barclay C, Dahlhoff EP (2007). Phosphoglucose isomerase genotype affects running speed and heat shock protein expression after exposure to extreme temperatures in a montane willow beetle. J Exp Biol.

[16] Sambe MA, He X, Tu Q, Guo Z (2015). A cold-induced myo-inositol transporter-like gene confers tolerance to multiple abiotic stresses in transgenic tobacco plants. Physiol Plant.

[17] Bentley DR (2006). Whole-genome re-sequencing. Curr Opin Genet Dev.

[18] Irizarry RA, Warren D, Spencer F, Kim IF, Biswal S, Frank BC (2005). Multiple-laboratory comparison of microarray platforms. Nat Methods.

[19] Pedotti P, t Hoen PA, Vreugdenhil E, Schenk GJ, Vossen RH, Ariyurek Y (2008). Can subtle changes in gene expression be consistently detected with different microarray platforms?. BMC Genomics.

[20] t Hoen PA, Ariyurek Y, Thygesen HH, Vreugdenhil E, Vossen RH, de Menezes RX (2008). Deep sequencing-based expression analysis shows major advances in robustness, resolution and inter-lab portability over five microarray platforms. Nucleic Acids Res.

[21] Wilhelm BT, Landry JR (2009). RNA-Seq-quantitative measurement of expression through massively parallel RNA-sequencing. Methods.

[22] Velculescu VE, Kinzler KW (2007). Gene expression analysis goes digital. Nat Biotechnol.

[23] Licatalosi DD, Darnell RB (2010). RNA processing and its regulation: global insights into biological networks. Nat Rev Genet.

[24] Sorek R, Cossart P (2010). Prokaryotic transcriptomics: a new view on regulation, physiology and pathogenicity. Nat Rev Genet.

[25] Metzker ML (2010). Sequencing technologies—the next generation. Nat Rev Genet.

[26] Huang W, Marth G (2008). EagleView: a genome assembly viewer for next-generation sequencing technologies. Genome Res.

[27] Morozova O, Marra MA (2008). Applications of next-generation sequencing technologies in functional genomics. Genomics.

[28] Cloonan N, Grimmond SM (2008). Transcriptome content and dynamics at single-nucleotide resolution. Genome Biol.

[29] Wang Z, Gerstein M, Snyder M (2009). RNA-Seq: a revolutionary tool for transcriptomics. Nat Rev Genet.

[30] Anisimov SV (2008). Serial Analysis of Gene Expression (SAGE): 13 years of application in research. Curr Pharm Biotechnol.

[31] David JP, Coissac E, Melodelima C, Poupardin R, Riaz MA, Chandor-Proust A (2010). Transcriptome response to pollutants and insecticides in the dengue vector Aedes aegypti using next-generation sequencing technology. BMC Genom.

[32] Zhang Y, Jiang R, Wu H, Liu P, Xie J, He Y, Pang H (2012). Transcriptome profiling analysis of insecticide stress Cryptolaemus montrouzieri reveals resistance-relevant genes in ladybird. Genomics..

[33] Pan Q, Shai O, Lee LJ, Frey BJ, Blencowe BJ (2008). Deep surveying of alternative splicing complexity in the human transcriptome by high-throughput sequencing. Nat Genet.

[34] Mattick JS (2009). The genetic signatures of noncoding RNAs. PLoS Genet.

[35] Audic S, Claverie JM (1997). The significance of digital gene expression profiles. Genome Res..

[36] Hanriot L, Keime C, Gay N, Faure C, Dossat C, Wincker P (2008). A combination of LongSAGE with Solexa sequencing is well suited to explore the depth and the complexity of transcriptome. BMC Genom.

[37] Georg RC, Gomes SL (2007). Transcriptome analysis in response to heat shock and cadmium in the aquatic fungus Blastocladiella emersonii. Eukaryot Cell.

[38] Zeng T, Li JJ, Wang DQ, Li GQ, Wang GL, Lu LZ (2014). Effects of heat stress on antioxidant defense system, inflammatory injury, and heat shock proteins of Muscovy and Pekin ducks: evidence for differential thermal sensitivities. Cell Stress Chaperones.

[39] Gleason LU, Burton RS (2015). RNA-seq reveals regional differences in transcriptome response to heat stress in the marine snail Chlorostoma funebralis. Mol Ecol.

[40] Sun L, Lamont SJ, Cooksey AM, McCarthy F, Tudor CO, Vijay-Shanker K (2015). Transcriptome response to heat stress in a chicken hepatocellular carcinoma cell line. Cell Stress Chaperones.

[41] Morrissy AS, Morin RD, Delaney A, Zeng T, McDonald H, Jones S, Zhao Y, Hirst M, Marra MA (2009). Next-generation tag sequencing for cancer gene expression profiling. Genome Res..

[42] Eisen MB, Spellman PT, Brown PO, Botstein D (1998). Cluster analysis and display of genome-wide expression patterns. Proc Natl Acad Sci USA.

[43] Saldanha AJ (2004). Java Treeview—extensible visualization of microarray data. Bioinforma..

